RETRACTED

# Action Recognition Model in Choral Conducting Teaching in Colleges and Universities under New Media Environment

**DOI:** 10.1155/2022/9330699

**Published:** 2022-08-11

**Authors:** Jian Jiao

**Affiliations:** Lanzhou University of Finance and Economics, Lanzhou City, Gansu Province, China

## Abstract

In current college music education, choral conducting is a required course for students. The course implementation aims to cultivate excellent and high-quality choral conductors. The requirements for choral conducting teaching in college music education under the new media environment have been further improved. First, this study gives the value of applying new media technology in choral conducting teaching in colleges and universities. Then, based on the key point that choral conductors' expression of music mainly relies on gestural language, an action recognition model in college choral conducting teaching is proposed. The model is designed with an adaptive deep graph convolution model, and a spatio-temporal convolution submodel with a small number of parameters is created using group convolution. After the trained teacher model is obtained, the spatio-temporal convolutional submodel with fewer parameters is trained using the knowledge distillation method combined with data augmentation techniques. The final action recognition fusion model is obtained using the linear fusion method. The experimental results demonstrate that the proposed model can recognize the movements in college choral conducting teaching with higher performance than other existing models, which provides effective guidance for college choral conducting teaching in the new media environment.

## 1. Introduction

The special nature of the art of choral singing has led most music education majors in colleges and universities to emphasize teaching choral conducting. As a basic course for college music education students, choral conducting is also one of the courses teaching with the highest application rate for students to engage in music-related education work in the future [1]. Great importance should be attached to the rationality of the teaching mode of music education majors in colleges and universities and choral teaching and rehearsals are organized in schools to provide sufficient guarantee for future music education talents [2]. China's national comprehensive music literacy choral art development is relatively weak, mainly because of the lack of excellent conductor talents. The number is relatively insufficient. The reform of the choral conducting education curriculum for college music majors needs to be put into practice to help the curriculum of choral conducting for college music majors to be more scientific and rationalized and cultivate more excellent talents for the country [2, 3].

RETRACTED

The choral conductor is the creator of the art of collective singing [4, 5]. For the conductor, his task is not only to play the beat but also to read through the whole work before conducting the performance and to savor the emotions to be expressed in each stage of the score. After a profound analysis of the work, gestures were designed in advance to convey the professional singing players, with the choir voice to compose the real emotional color of the musical work [6].

The new media environment has provided good channels and methods for teaching choral conducting in colleges and universities [7, 8]. Some teachers have been trying to introduce the Internet and new media technology into the classroom, but a systematic teaching system has not yet been formed. On the one hand, the new media teaching facilities in colleges and universities are not completely popular. Many colleges and universities are not equipped with new media teaching equipment and promotion platforms. On the other hand, teachers lack operating experience and have not built cooperation relationships with Internet-related enterprises. Therefore, college teachers should use the resources and platforms in the new media era and integrate new scientific technologies (such as movement recognition technology) into the teaching classroom. This can explore the new modern choral conducting teaching mode, find more powerful support, and open up a broader space for innovation to improve the teaching practice effect.

Action recognition is a fundamental task in computer vision and has many applications in security, medical, and sports fields [9]. Early on, people mainly studied action recognition based on RGB data, depth data, optical flow data, etc. With the improvement of the accuracy of human pose and key point estimation by deep learning techniques, many tools and devices have been spawned. They can easily estimate human skeleton data, which has attracted many researchers to study skeleton-based action recognition. The skeleton is a simple representation of the human body structure and pose, and each frame of skeleton data contains multiple key points (joints). The skeleton data of different moments are combined to form a skeleton series representing an action. Skeleton data are widely used in human action recognition because of their simplicity, less redundant information, and fast computation.

Literature [10] uses support vector machines and K-means clustering methods to classify actions. Such traditional machine learning-related algorithms require the manual design of classification features with weak expressiveness. They are incapable of classification tasks with many classification categories and large datasets. The deep learning class can be divided into RNN class methods [11], GCN class methods, and other CNN class methods, and the most researched RNN class methods use long short-term memory (LSTM) structure to solve the problem. Models containing different LSTM variants, such as ST-LSTM (spatio-temporal long short-term network) [12] and part-aware LSTM, have been designed by previous authors. Models with LSTM structure are prominent in tasks dealing with temporal data classes such as speech and text. However, the skeleton data here can also be considered time-series data. The difference is that there is a strong reliance on the variation of the skeleton data in all dimensions of space and time in action recognition. This makes it difficult for the LSTM method to take advantage of its ability to handle time-series data. Other CNN-like methods, such as two-stream 3D CNN with 3-dimensional convolution, are available [13]. We can arrange the skeleton data in different ways and design customized convolutional kernel sizes to meet the 2-dimensional convolutional operation, such as TCN (temporal convolutional networks) and synthesized CNN. However, because the key points of the skeleton are naturally connected in the human body, a common shortcoming of these methods is that they do not make good use of the “intrinsic information” of the skeleton data. In addition, one of the obvious disadvantages of other methods that use 3D convolution is that 3D convolution leads to a large number of model parameters and high computational cost. GCN has been one of the most used methods in this problem in the last two years [14].

RETRACTED

The GCN-like approach can explicitly represent the spatial location relationship of key points, such as the adjacency matrix, and design the update method of data in the model based on the spatial topological relationship and time-domain information. Compared with other methods, the GCN-like approach achieves better results on multiple datasets and is more suitable for the task of action recognition based on skeleton key points. At present, many cutting-edge GCN-like methods have complex model structures with deep layers and many parameters. Therefore, there is a need to study simpler, lighter, and more robust models. In addition, the coordinates of key points, angles, and camera views are important information, and different forms of input data have a significant impact on the model accuracy. The ST-GCN model is the first to apply graph-based convolutional networks to skeleton-based action recognition [15]. Literature [16] adds an attention (attention) module to the graph convolutional network layer to help the network pay more attention to the input data's important points, frames, and features. In literature [17], a new dual-stream graph convolution model is designed, which better learns the valid information in both time and space domains.

RETRACTED

This study proposes an improved adaptive deep graph convolution model based on the existing research. The model decouples the node representation transformation and the feature propagation and adds initial residuals to the feature propagation process of the nodes. Then, the node representations obtained from different propagation layers are combined adaptively. The appropriate local and global information is selected for each node to obtain an information-rich node representation. A small number of labeled nodes are used for supervised training to generate the final node representation. Finally, a spatio-temporal convolutional submodel with few parameters is trained using a knowledge distillation approach combined with data augmentation techniques.

This study has four main innovations and contributions:

1. The initial residuals and decoupling operations are jointly applied to the graph convolutional network, and an adaptive mechanism obtains the final node representation.
2. A lightweight temporal convolution module is designed using group convolution and other techniques to reduce the number of model parameters. For the first time, knowledge distillation is applied to the action recognition problem based on skeleton data to ensure the model's accuracy after the parameter quantity is reduced.
3. Data augmentation techniques such as affine transformation are used to add new forms of input data to the model, which adds additional perspectives for observing the action and increases the robustness of the model.
4. A parallel fusion model with multiple strands is proposed with higher recognition accuracy on the dataset.

This study consists of four main parts: the first part is the introduction, the second part is the methodology, the third part is the result analysis and discussion, and the fourth part is the conclusion.

## 2. Methodology

### 2.1. Choral Conducting Teaching in Colleges and Universities under the New Media Environment

#### 2.1.1. Create a New Learning Environment That Is Different from the Traditional Teaching Classroom

The ubiquitous spread and coverage of new media have greatly changed the college choral conducting teaching environment and put forward higher requirements for college choral conducting teaching. The traditional choral conducting teaching mode is no longer well adapted to the current new media environment. In the mobile new media environment, with the help of new media technology innovation, choral observation teaching lets students intuitively experience the development of new ideas of choral conducting teaching and jointly broadens the vision of choral conducting teaching for teachers and students. Teachers in colleges and universities should combine theoretical knowledge with modern technology to create a new effective learning environment different from the traditional teaching classroom. They should guide students to take the initiative to use modern technology to plan their learning plans, use big data to summarize and monitor their learning process in the learning process, and make a reflective evaluation of their learning effectiveness.

RETRACTED

With the rapid development of technology, new media means of teaching choral conducting in colleges and universities have provided many facilities for teaching. The new media of choral video images create an infinite loop of learning self-examination environment for teachers and students, as shown in Figure 1. This ability helps students remove themselves from the complexity of the phenomena and stand on an equal footing to observe together. Choral works ultimately display different cultures and a presentation of life beliefs. Therefore, college teachers should fully consider the value and role of new media in classroom teaching, create a high-quality new learning environment, and quickly realize all-around communication between offline and online teaching. They integrate various levels of teaching tools to make the choral course content colorful. Teachers and students can experience the cultural connotation of choral art and understand the synchronization of the choral profession with the trend of music development in the learning process, thus enhancing the effectiveness of their teaching innovation.

#### 2.1.2. Build a Good Environment for Music Listening Experience

Through the trend of today's technological development, the music of different cultures, styles, and genres from all over the world is brought together by using the new media information transmission with wide coverage and fast speed. Teachers and students listen together to the experiences of outstanding former choral training and enjoy the exhibition of outstanding choral groups. This will guide students to engage in the activity of listening with multiple senses. In the music listening environment, the musical elements are concretized and visualized. A choral sound that combines flat and three-dimensional elements is built. The horizontal and vertical harmonic lines are understood. The integration of musical melody and conducting gestures is experienced. A choral music mindset that is ready for analysis is ultimately developed.

RETRACTED

The quick and easy access to the new media age provides students with many types of choral music pieces to appreciate. Music listening skills are deepened and the music is connected to the students' hearts. It also allows students to record and listen to their conducting singing, evaluate each other's or other students' singing or conducting, and offer their own opinions and suggestions. The previous teacher-led traditional model is changed and a new student-oriented teaching atmosphere is created.

#### 2.1.3. Innovative Measures for Teaching Choral Conducting in Colleges and Universities in the New Media Era

A two-year professional study plan is planned for students. With students as the main learning subjects, their learning success is recorded at different stages in video format. This allows us to find the trajectory of students' learning progress, adjust the teaching progress in real time, and revise the teaching plan.

In 2020, the online choral conducting lecture series and “cloud choral” performance activities launched by various universities had filled the regret of not being able to listen to the lectures of conducting experts and excellent team singing due to the epidemic. During the epidemic, some teachers used the new media technology platform to forward the learning content to students in advance by employing video. Students directly observed and studied the integrated rehearsal methods used by the best conductors. This prompts students to generate feedback and deepen their understanding of music learning. They also use new media technology materials to supplement their teaching and find motivation for continuous improvement by observing their conducting videos at different stages of learning.

In a new media environment, teachers incorporate new scientific technologies (such as motion recognition technology) into the classroom to build a diverse teaching model that equips students with the ability to continuously acquire musical experiences.

### 2.2. Action Recognition Model

#### 2.2.1. Adaptive GCN

This section will first give the original formulation of the two-layer graph convolution as shown in the following formula:

(1) $$\begin{array}{c} K=\text{softmax}\left(\hat{G}\text{ReLU}\left(\hat{G}IM^{\left(0\right)}\right)M^{\left(1\right)}\right), \end{array}$$

where $\hat{G}={\hat{D}}^{-1/2}\hat{G}{\hat{D}}^{-1/2}$. First, the original identity matrix *I* is transformed by the transformation matrix *M*. Then, matrix operations are performed with the symmetrically normalized adjacency matrix $\hat{G}$. Finally, a nonlinear activation function is applied. The previous layer's output is used as the input of the next layer.

RETRACTED

Formula (1) shows that the feature propagation and transformation are coupled together during the graph convolution, which makes the model's training difficult when deep graph convolution is performed. In this study, an improved adaptive graph convolution network is proposed. The network model is based on a graph convolutional neural network with the removed nonlinear activation function and transformation matrix. It applies the initial residuals and decoupling operations to the graph convolutional network and obtains the final node representation by an adaptive mechanism.

To understand the feature propagation and representation transformation in coupled graph convolution, the model proposed in this study first processes the original representations of the nodes using a multilayer perceptron to generate representations for subsequent propagation. These representations contain only information about the nodes themselves, no structural information. The dimensionality is much smaller than the initial feature dimensionality of the nodes, which is exemplified here by the *x*th node, as shown in the following formula:

(2) $$\begin{array}{c} b_{x}^{0}=\text{MLP}\left(I_{x}\right)\in R^{c}, \end{array}$$

where *b*_*x*_^0^ is the node representation obtained by dimensionality reduction of the multilayer perceptron. *c* indicates the number of node categories.

The structural information of the graph is integrated into the node representation during the propagation process. As the number of propagation layers gradually increases, the percentage of information of the nodes themselves will gradually decrease. The method in this study utilizes an initial residual connection in the propagation process to further preserve the information of the nodes themselves. In this way, even if many layers are propagated, the generated node representation still retains part of the node information as shown in the following formulas (3) and (4):

(3) $$\begin{array}{c} b_{x}^{\ell^{\prime }}=\sum_{y\in T\left(q_{x}\right)}\frac{1}{\sqrt{\left|T\left(q_{x}\right)\right|}\sqrt{\left|T\left(q_{y}\right)\right|}}b_{y}^{\ell -1}, \end{array}$$

(4) $$\begin{array}{c} b_{x}^{\ell }=\left(1-\alpha \right)b_{x}^{\ell^{\prime }}+\alpha b_{x}^{0}, \end{array}$$

where *b*_*x*_^*ℓ*^ is the representation obtained by propagating node *q*_*y*_ through *ℓ* layers. *T*(*q*_*y*_) denotes the set of neighbors of node *q*_*y*_. *α* denotes the residual retention rate. *ℓ*=1,2,…, *z*. *z* denotes the number of graph convolution layers.

However, it is difficult to determine an appropriate number of layers for propagation. Too few layers will not obtain sufficient and necessary information about the neighbors, and too many layers will bring too much global information, thus eliminating specific local information. The ideal most suitable receptive domain is different for each node. The representations obtained from different propagation layers have different degrees of influence on the final representations of the nodes. A learnable vector *p*_*x*_ is used in this study to compute the node representations obtained from different propagation layers to obtain the retention fractions of the corresponding representations. These retention scores measure how much of the information of the corresponding representations generated by the different propagation layers should be retained.

(5) $$\begin{array}{c} p_{\ell }=p_{x}^{N}b_{x}^{\ell }, \end{array}$$

where *p*_*ℓ*_ indicates the reservation fraction of the representation obtained by convolution of the *ℓ*-layer map.

RETRACTED

The different propagation layers' representations are weighted and summed to obtain the final node representation as shown in the following formula:

(6) $$\begin{array}{c} k_{x}=\sum_{\ell =0}^{z}p_{\ell }b_{x}^{\ell }, \end{array}$$

where *k*_*x*_ is the final representation of node *q*_*y*_ used for prediction.

Using this adaptive adjustment mechanism, the model can achieve an adaptive balancing of the information of local and global neighborhoods of each node. The overall framework of adaptive GCN is shown in Figure 2.

The single node is updated in a way that matrix operations are used here to facilitate multiple node updates:

(7) $$\begin{array}{c} B_{0}=\text{MLP}\left(I\right)\in R^{T\times c}. \end{array}$$

Here, *B*_0_ denotes the representation matrix used for propagation. It is obtained from the initial node representation matrix *I* after passing through a multilayer perceptron:

(8) $$\begin{array}{c} B_{\ell }=\left(1-\alpha \right){\hat{G}}^{\ell }B_{0}+\alpha B_{0}\in R^{T\times c}, \end{array}$$

where *B*_*ℓ*_ denotes the representation matrix of the nodes at layer *ℓ*.

(9) $$\begin{array}{c} B=\text{stack}\left(B_{0},B_{1},\text{…},B_{z}\right)\in R^{T\times \left(z+1\right)\times c}. \end{array}$$

The representation matrices obtained from different propagation layers are stacked using stack operations to obtain the representation matrix *B*. This representation matrix is used for the subsequent calculation of the retention fraction:

(10) $$\begin{array}{c} P=\sigma \left(Bp\right)\in R^{T\times \left(z+1\right)\times 1}. \end{array}$$

A shared learnable vector *p* ∈ *R*^*c*×1^ is used to compute the retention fractions of different propagation layer representations to obtain the retention fraction matrix *P*:

(11) $$\begin{array}{c} \hat{P}=\text{reshape}\left(P\right)\in R^{T\times 1\times \left(z+1\right)}, \end{array}$$

where $\hat{P}$ is obtained by dimensionally transforming the retention score matrix *P* using the reshape operation.

(12) $$\begin{array}{c} K=\text{softmax}\left(\text{squeeze}\left(\hat{P}B\right)\right)\in R^{T\times c}. \end{array}$$

Dimensionality compression is performed using the squeeze, and normalization operation is performed with softmax to obtain the representation matrix *K* of the nodes used for prediction.

RETRACTED

#### 2.2.2. Action Recognition Model

Model fusion is a strategy used in various fields of deep learning, which aims to fuse some branching networks with weak expressiveness to build a globally optimized overall model. In the problem of skeleton-based action recognition, a graph convolution is an effective approach. However, different structures of graph convolution models extract different features, and the models make recognition judgments based on different feature information. The fusion models can be used to complement each other.

The overall schematic diagram of the model is presented in Figure 3. The fusion model consists of a DGC submodel and an AGC submodel. The temporal convolution module uses a grouped convolutional design with a small number of submodels.

*(1) DGCNNet*. DGCNNet is a submodel of the fusion model proposed in this study, which contains ten layers of light-DGC base layers, as shown in Figure 4. The dashed box indicates the convolution when the number of channels of the current post-tensor does not match. In this study, the following design is carried out in the light-DGC base layer:

1. The self-attention module is cascaded after the spatial convolution module. In deep learning neural networks, self-attention is a mechanism used to calculate the importance of features at different input data locations. Each self-attention module learns a weight tensor to represent the “importance” of each feature at each location. This mechanism has been successfully applied to various tasks in speech recognition, text translation, and computer vision. Three self-attentive modules are cascaded after the spatial convolution module to learn a coefficient vector for each of the three dimensions of the feature map: temporal, spatial, and feature, which is used to enhance the impact of important points, important frames, and important feature channels in the feature map on the model classification.

The self-attention mechanism (SAM) was originally proposed by Vaswani in 2017. They detailed the principle of SAM and the transformer language translation model constructed based on this mechanism in the literature. The calculation of self-attention is shown in Figure 5.

RETRACTED

Taking a sequence of 4 vectors {*g*_1_, *g*_2_, *g*_3_, *g*_4_} as an example, we next calculate the attention scores of each of these 4 items. First, given the parameter matrices *M*^*v*^, *M*^*z*^, *M*^*q*^ (whose values are determined by training), *g*_*i*_ is multiplied with each of the three matrices to obtain *v*_*x*_, *z*_*x*_, *q*_*x*_, where *x*=1,2,3,4. Then, the inner product of *v*_*x*_ and *z*_*y*_ is obtained as *α*_*xy*_, where *x*, *y*=1,2,3,4. The matrix *α*_*xy*_ is normalized to obtain the matrix ${\hat{\alpha }}_{xy}$, which is the attention score matrix. Finally, $h_{x}=\sum_{y=1}^{4}{\hat{\alpha }}_{xy}\cdot q_{x}$ is taken as the output of the self-attentive mechanism with *x*=1,2,3,4.

From the computational approach, it can be seen that the purpose of the self-attentive mechanism is to assign the information of all input items in the sequence to each of them. That is, each input item can be inferred using the information of the whole sequence, thus ensuring that the deep learning model can use contextual information to classify the input sequence. When processing sequence information, recurrent neural network (RNN) is a temporal logic that relates contextual information by repeating the state transfer on the module. The self-attentive mechanism shares the information of all the input items simultaneously by a set of operations, which results in shorter processing steps and more comprehensive information sharing.

(2) To learn the temporal variation information better, the convolution kernel of the time domain dimension is usually larger. The use of normal convolution leads to more parameters in the model. Therefore, the light-TCN module, which is used to update the time-domain information of the data, uses a grouped convolution with a smaller number of parameters instead of the normal full convolution. The light-TCN module uses a channel-by-channel 2-dimensional convolution with a convolution kernel of (1) and (9) and a normal 2-dimensional convolution with a kernel of (1) and (1) to process the time-domain information of the feature map, replacing the normal 2-dimensional convolution with a convolution kernel of (1) and (9). After using grouped convolution strategy, the number of input and output feature map channels is denoted by *C*_*x*_ and *C*_*o*_, respectively. The number of parameters in this module is reduced from *C*_*o*_ × *C*_*x*_ × 9 × 1 to *C*_*o*_ × 1 × 1 × 9+*C*_*o*_ × *C*_*x*_ × 1 × 1 when only the convolution is considered.

*(2) AGCNNet*. The adjacency matrix is used to represent the connection relationship between the key points of the human skeleton, and the convolution method is set based on the connection relationship. The data of each point are updated by the points connected to it, which is another type of widely used graph convolution model. In order to be able to pay more attention to important frames, important points, and important features during model training, this study uses adaptive graph convolution as the spatial convolution module of the model to build the fusion model AGCNNet, which consists of 10 light-AGC base layers. The light-AGC base layer is shown in Figure 6. The dashed box indicates the use of convolution when the current post-tensor channel number does not match. The light-AGC base layer updates the time-domain information of the feature map using the light-TCN module with fewer parameters than other existing methods.

*(3) Knowledge Distillation Model Training*. Knowledge distillation can transfer the knowledge learned from the complex model in the same task to the simple model and improve the expressiveness of the simple model, thus achieving the purpose of using the simple model to deal with complex problems. The distillation training method used in this study is shown in Figure 7. The training process is divided into two steps:

(1) Train a teacher model using the training data and save the model's parameters.
(2) The features before the fully connected layer of the teacher model are used as “privileged information.” Combine with the training data to train the student model, use *fc*_tea_ to represent the “privileged information” feature layer of the teacher model, and use the mean squared error (MSE) of the corresponding feature layer *fc*_stu_ of the student model as one of the loss functions. Together with the cross entropy between the model prediction $\hat{J}$ and the data label *J*, they form the final loss function. A weighting factor *β* of the mean squared error term is added to the loss function to adjust the weight of the mean squared error term. The final loss function for training is as follows:
  (13) $$\begin{array}{c} L=\text{cross Entropy}\left(\hat{J},J\right)+\beta \times \text{MSE}\left(fc_{\text{tea}},fc_{\text{stu}}\right), \end{array}$$

where crossEntropy ( ) denotes the calculation of cross entropy loss and MSE() denotes the calculation of mean squared error loss.

RETRACTED

For distillation training, DGCNNet and AGCNNet models were used as student models. AGCN and DGNN were used as distillation training submodels for the teacher model. The effectiveness of the distillation training method used was demonstrated by comparing the accuracy of the student model with that of the teacher model.

*(4) Data Enhancement*. Various kinds of augmented data have been used in previous studies, among which motion data are widely used to improve accuracy. However, in general, the model's accuracy is low when the motion data are trained alone. In this study, we choose affine transformation as the data augmentation method. The skeleton data after affine transformation are used as augmented data to improve the robustness of the model to different viewpoints. In the NTU RGB + D dataset, the key points of human body joints are points in 3-dimensional space, and the coordinate values of the vertical axis with the ground are kept unchanged during the data transformation. The affine transformation is applied to the coordinate values in other dimensions. For the key point *I*, after affine transformation, the transformed data *I*_*g*_=*I* · *G*+*h* are obtained, where, $G=\left(\begin{array}{ccc} \text{cos}\varphi & -\text{sin}\varphi & 0\\ \text{sin}\varphi & \text{cos}\varphi & 0\\ 0 & 0 & 1 \end{array}\right)$.

*(5) Model Fusion*. The input of DGCNNet includes two forms, namely, skeleton data (joints + bone) and skeleton data after affine transformation, because the input form of data is increased by using affine transformation. The input of AGCNNet includes joints, bone, affine transformed joints, and affine transformed bone in four forms. Using the distillation training method, six submodels with a small number of parameters are trained. In the final test, the output of the softmax function of the submodels is summed up as the final output. The output of the softmax function of the *x* th submodel is denoted by ${\hat{J}}_{x}\left(x=1,\text{…},6\right)$, and the final prediction value is as follows:

(14) $$\begin{array}{c} \hat{J}=\sum_{x=1}^{6}{\hat{J}}_{x}. \end{array}$$

## 3. Result Analysis and Discussion

### 3.1. Dataset

This study uses two datasets for the experiments:

Dataset 1 is the NTU-RGBD dataset. This dataset is currently the largest indoor dataset for action recognition. It contains 56880 data samples from 60 categories. Each category contains data of 40 volunteers captured by 3 Kinect v2 cameras. The following two subsets can be obtained according to different partitioning criteria: cross-subject (CS) and cross-view (CV). *Cross-Subject (CS)*: the dataset is partitioned according to the number of volunteers. The training set has 40320 samples and the test set has 16560 samples. *Cross-View (CV)*: the dataset is divided according to the camera number. The training set has 37,920 samples, and the test set has 18,960 samples.

Dataset 2 is a dataset of conducting gestures intercepted through choral conducting videos. There is no database of choral conducting gesture images. In this study, the collected sample data are processed. The obtained conducting action data are used as the experimental database. The conducting database contains 20 basic gestures. There are 100 images for each gesture, totaling 2,000 gesture images. The size of each image is 148∗148.

RETRACTED

### 3.2. Parameter Setting

The experimental environment is Windows 10, the CPU is Intel(R) Core(TM) i7-9750H, the GPU is GeForce GTX 1650, and the design network is implemented using PyTorch deep learning framework. For DGCNNet and AGCNNet subnetworks, the models are built using a 10-layer light-DGC base layer and a 10-layer light-AGC base layer. The number of output channels is the same for both subnetworks. Ten-layer output channels are 64, 64, 64, 64, 64, 128, 128, 128, 256, and 256, respectively. The training data batch size is 32. The optimizer uses stochastic gradient descent (SGD). The learning rate was initialized to 0.1.

When training the teacher network, the learning rate was reduced to 1/10 after 40 and 90 generations, and the model was trained for a total of 120 generations. When training the student network, the learning rate was reduced to 1/10 after 30 and 40 generations. For distillation training, the value of *β* in the loss function was determined experimentally. The AGCN model with pretrained and fixed weights was used as the teacher model, and AGCNNet was used as the student model for training and testing the bone data. The different values of *β* and the corresponding test accuracy are shown in Figure 8. According to the experimental results, the *β* values of distillation training for all submodels were set to 50.

### 3.3. Adaptive GCN Performance

The proposed model is compared with other models to verify the performance of the adaptive GCN proposed in this study. The comparison models are GCN, graph attention network (GAT), simplifying graph convolutional network (SGC), PageRank-GCN [18], and DAGNN [19]. The recognition results of different models are given in Figure 9.

As can be observed from Figure 9, the classification effectiveness of adaptive GCN on dataset 2 is improved by 6.6 percentage points compared to GCN, demonstrating the superiority of the model in this study for the semisupervised node recognition task on the dataset.

### 3.4. Student Model Vs. Teacher Model

The student model uses a lightweight temporal convolution module, significantly reducing the model parameters. The model distillation training method is also used to make the model have high accuracy with fewer parameters. For the DGC-NNet submodel, the DGNN is first trained on the skeleton data joints + bone, and then the student model DGCNNet is trained by distillation of the model. The distillation results of the AGCNNet and DGCNNet student models were compared with the corresponding teacher models in terms of the number of parameters and accuracy, as shown in Figure 10.

RETRACTED

The results in Figure 10 indicate that the number of parameters of the student models for both structures was significantly reduced (by about 50%). The accuracy of the model trained by distillation is higher than that of the one without distillation training and even higher than that of the teacher model with a large number of parameters. It is due to using a lightweight time-domain convolution module in the student model, which reduces the number of parameters. Moreover, the constraints from the teacher model are increased by the loss function during training, and the recognition accuracy of the student model is ensured by using the model distillation training method.

### 3.5. Performance Analysis of the Fusion Model

It was compared with other frontier methods [20–24] on the choral command dataset to verify the performance of the fusion model proposed in this study. The comparison results are shown in Figure 11.

The results in Figure 11 demonstrate that the model's accuracy in this study reached 96.6% on the dataset, respectively, which is significantly better than the benchmark method based on ST-GCN in literature [15] with 88.4%. Compared with other excellent frontier methods, it is also relatively competitive. This is because, first, the model in this study uses initial residual connectivity and decoupled graph convolution networks to improve the original graph convolution and uses an adaptive mechanism to integrate the node representations of different propagation layers. Through distillation learning, a lightweight time-domain convolution module is used in the student model, which reduces the number of parameters of the model. Moreover, the constraints from the teacher model are increased by the loss function during training, and the recognition accuracy of the student model is ensured by using the model distillation training method. Finally, the affine transformation for data augmentation can further help the model improve accuracy.

## 4. Conclusion

The integration of new media technology in choral conducting teaching in colleges and universities is one of the important means to innovate choral conducting teaching. Therefore, college teachers need to fully explore the application mode of integrating new media technology and artificial intelligence technology with traditional teaching in the future teaching process. In this study, under such a requirement, an action recognition model of choral conducting teaching in colleges and universities under the new media environment is proposed. The model is first designed with adaptive GCN. Then, a spatial convolution module is constructed with two different structures of graph convolution, combined with self-attentive modules in 3 dimensions such as channel, space, and time. A multibranch lightweight submodel is constructed using a temporal convolution module designed with group convolution on a channel-by-channel basis. The distillation training method is used to distill knowledge from the teacher model with many parameters to train these student submodels. Data augmentation techniques such as affine transformations are used to augment the input data during training and testing to increase the robustness of the models. Eventually, the training resulted in lighter and more accurate submodels.

RETRACTED

Further, a multistranded parallel fusion model with a smaller number of parameters and better accuracy and robustness was constructed by fusing them. The experimental results indicate that the model's accuracy is greatly improved compared to the graph convolution approach and outperforms many existing skeleton-based action recognition frontier algorithms. In future work, it is proposed to investigate the problem of action recognition for choral conducting with small variations. Such action recognition is closely related to the environment and surrounding objects. It requires using other data such as RGB data combined with techniques such as object detection and recognition to construct a graph of the relationship between the person and the environment and surrounding objects.

## Figures and Tables

**Figure 1:** The learning self-checking environment in commanding teaching.

**Figure 2:** Overall framework of adaptive GCN.

**Figure 3:** Schematic diagram of the fusion model.

**Figure 4:** Light-DGC layer.

**Figure 5:** Self-attention calculation method.

**Figure 6:** Light-AGC layer.

**Figure 7:** Model distillation training.

**Figure 8:** The model accuracy.

**Figure 9:** Recognition accuracy.

**Figure 10:** Performance comparison of student model and teacher model.

**Figure 11:** Identification results of proposed model and other existing models.

## Data Availability

The labeled dataset used to support the findings of this study is available from the corresponding author upon request.
